The article "Multitask Healthcare Management Recommendation System Leveraging Knowledge Graph" was published in 2021. Journal: J Healthc Eng.

# Multitask Healthcare Management Recommendation System Leveraging Knowledge Graph

**DOI:** 10.1155/2021/1233483

**Published:** 2021-11-05

**Authors:** Wanheng Liu, Ling Yin, Cong Wang, Fulin Liu, Zhiyu Ni

**Affiliations:** ^1^Beijing University of Posts and Telecommunications, Beijing, China; ^2^National Population Health Data Center, Changping, China; ^3^Affliated Hospital of Hebei University, Baoding, Hebei, China

## Abstract

In this paper, a novel multitask healthcare management recommendation system leveraging the knowledge graph is proposed, which is based on deep neural network and 5G network, and it can be applied in mobile and terminal device to free up medical resources and provide treatment programs. The technique we applied is referred to as KG-based recommendation system. When several experiments have been carried out, it is demonstrated that it is more intelligent and precise in disease prediction and treatment recommendation, similar to the state of the art. Also, it works well in the accuracy and comprehension, which is much higher and highly consistent with the predictions of the theoretical model. The fact that our work involves studies of multitask healthcare management recommendation system, which can contribute to the smart healthcare development, proves to be promising and encouraging.

## 1. Introduction

Recently, intelligent healthcare recommendation system has become a hot topic in healthcare management application research. As much attention has been paid to health, people have been gradually changing from the passive response to medical treatment to the active normal prevention and performing healthcare. Driven by the need for healthcare management application, an accurate and efficient healthcare recommendation system which can be applied in terminal device is now playing an important role in healthcare, which not only can make a more comprehensive and continuous record and analysis of our health condition but also can recommend appropriate health interventions and treatment programs. It can contribute to freeing up more medical resources while improving efficiency and accuracy.

It is known that the traditional recommendation system is to solve the problem of information explosion and there are two major tasks in it, including rating prediction and CTR prediction. Previously, most of the studies on recommendation system focused on collaborative filtering [1], content-based filtering [2], and hybrid method [3]. Collaborative filtering algorithm starts from similarity measurement to consider the similarity between users or items to make recommendations; and content-based recommendation methods can learn the representation of user and item form the contents of item. However, hybrid method is designed to address the problem of cold start and sparsity in the interaction matrix data. It can combine content information of the user and the item for integration into the collaborative filtering framework to obtain better performance.

The article "Multitask Healthcare Management Recommendation System Leveraging Knowledge Graph" was published in 2021. Journal: J Healthc Eng.

While traditional recommendation system has made great progress, the accuracy and the explainability of the system are still the problem that needs to be solved. To fill the gaps, KG-based recommendation systems were carried out, in which the knowledge graph served as auxiliary information to be integrated into the recommendation system to improve the precision, diversity, and explainablity in it. The approaches of KG-aware recommendation system can be divided into three general classes: embedding-based method [4–7], path-based method [8, 9], and the unified method [10, 11]. The embedding-based method is to learn a low-dimensional feature for each entity and each relation in knowledge graph. In literature, Zhang et al. [4] in 2016 proposed using the heterogeneous information in knowledge to promote the quality of the recommendation system. In 2017, Wang et al. [5] put forward signing heterogeneous information network embedding for sentiment link prediction. Then, in 2018, they [6] presented a deep knowledge-aware network to integrate knowledge graph representation into news recommendation. Wang et al. [7] in 2019 proposed a multitask feature learning approach for knowledge graph enhanced recommendation. Besides, the basic idea of the path-based method is to design the connected similarity or the entity semantic similarity between user and item to improve the recommendations. In 2014, Xiao et al. [8] introduced metapath-based latent features to represent the connectivity between users and items. Hu et al. [9] came up with leveraging metapath-based context for top-N recommendation in 2018. Furthermore, the unified method is to combine the embedding method with the path-based method to fully excavate the information in both aspects. Wang et al. [10] in 2018 proposed RippleNetwork to incorporate the knowledge graph into recommendation system based on the unified method. In 2019, they raised Knowledge Graph Convolutional Networks (KGCN) [11], which is an end-to-end framework that captures interitem relatedness effectively by mining their associated attributes on the KG.

In addition, from the perspective of model structure, there are three forms in the combination of knowledge graph and recommendation system, sequential training [6], joint training [10], and alternate training [7]. Sequential training refers to the fact that the entity and relation vectors of the knowledge graph are obtained by embedding firstly. Then the recommendation system is introduced to learn the user vector and item vector for model training. In a word, it is conducted sequentially in the training of the embedding of the knowledge graph and the recommendation system. And joint training means that knowledge graph embedding and model training are simultaneous. What is more, in alternate training, it was trained alternately in the task of the feature learning in the knowledge graph and the click-through rate prediction of the model.

The article "Multitask Healthcare Management Recommendation System Leveraging Knowledge Graph" was published in 2021. Journal: J Healthc Eng.

As healthcare management in demand in our daily life and the recommendation system develops [12–14], Zaman et al. [12] proposed a personalized healthcare recommendation system using semantic web technology and healthcare social network in 2014. Also, Ahire et al. [14] in 2015 utilized the ontology based framework for healthcare recommendation system. Paramonov et al. [13] in 2016 also presented a recommendation service for smart space-based personalized healthcare system. Furthermore, it has become a tendency in healthcare management recommendation system which can be applied in mobile or terminal device to perform smart medical services. What is more, in literature, Archenaa et al. [15] presented health recommender system based on big data analytics in 2017. Guzmán et al. [16] in 2018 proposed a collaborative framework for sensing abnormal heart rate based on a semantic recommender system for healthcare. Meanwhile, Kaur et al. [17] proposed an efficient multiparty scheme for privacy preserving collaborative filtering for healthcare recommender system. Ali et al. [18] in 2018 presented a type-2 fuzzy ontology-aided recommendation system for IoT-based healthcare. Simultaneously, Somarathna et al. [19] proposed a recommendation system for customer preferred mental healthcare facility. Then Sahoo et al. [20] used collaborative filtering to perform deep learning based health recommender system in 2019. At the same time, Roy et al. [21] demonstrated integrating wearable devices and recommendation system toward a next-generation healthcare service delivery. Meanwhile, Rathi et al. [22] proposed a mobile based healthcare tool, an integrated disease prediction and recommendation system. In 2020, Noshad et al. [23] presented the clinical recommender system, which can predict medical specialty diagnostic choices with neural network ensembles. Simultaneously, Hussein et al. [24] proposed an accurate and reliable recommender system for chronic disease diagnosis. Meanwhile, Nagaraj et al. [25] designed a framework for e-healthcare management service based on recommender system. Then, in 2021, Ochoa et al. [26] raised a medical recommender system based on continuous-valued logic and multicriteria decision operators with interpretable neural networks. At the same time, Saad et al. [27] proposed a situation-aware recommendation system for personalized healthcare applications. Also, Pitchai et al. [28] presented a generic medicine recommendation system for advanced e-healthcare based on cloud computing. Meanwhile, Ponselvakumar et al. [29] proposed combining the recommendation system with deep learning to achieve the precision quality of healthcare. Moreover, to improve the performance of the recommendation system based on knowledge graph, in 2021, Andrea et al. [30] presented a comprehensive comparison of knowledge graph embedding-based link prediction methods. Meanwhile, Qian et al. [31] utilized a knowledge-aware multimodel adaptive graph learning principal for the effective feature learning. At the same year, Saikat et al. [32] proposed relation prediction of comorbid disease using knowledge graph completion of a tensor. In 2020, Huang et al. [33] provided a knowledge-driven multimodel activity recognition framework that exploits external knowledge to fuse multimodal data and reduce the dependence on large-scale training samples. In 2019, Wang et al. [34] proposed RippleNet, an end-to-end framework that naturally incorporates the KG into recommender systems.

The article "Multitask Healthcare Management Recommendation System Leveraging Knowledge Graph" was published in 2021. Journal: J Healthc Eng.

Great progress has been made in the performance of the recommendation system which can be applied in healthcare management, can improve the accuracy and the efficiency of the home visits and in treatment, and can also alleviate some medical resources. However, there are still some limitations in it: (1) Since the structural knowledge of the healthcare is the major information adopted in the knowledge base, it can be not comprehensive, precise, and efficient. (2) Due to single traditional recommendation system applied in healthcare management, it can lead to data sparsity, cold start problem, and overfitting. (3) Due to lack of abundant medical and healthcare data, the performance of the recommendation system is poor. (4) The deep neural network is not incorporated into most healthcare recommendation systems, which cannot lead to intelligence and efficiency to free up more medical resources and alleviate the pressure in treatment. (5) Owing to single disease paid attention to in the recommendation system, other diseases' prediction, diagnosis, and treatment recommendation would be ignored, which is incomprehensive.

In order to overcome the limitations and the problems above, a novel multitask healthcare management recommendation system leveraging the knowledge graph and deep neural network based on 5G network applied in mobile and terminal device is presented in this paper. To make it more comprehensive and accurate, except for the structural knowledge, the textual knowledge and the visual knowledge are also contained in the knowledge base. Then the knowledge graph is utilized in our healthcare recommendation to alleviate the problems of the single systems and be more precise and explainable. What is more, to acquire better performance, 600 thousand pieces of new data can be provided to support our system. In addition, deep neural network is also adopted in our system to make it more intelligent in various diseases' prediction, diagnosis, and treatment recommendation. Finally, it can be applied in mobile and terminal device, which can serve the patients and the doctors. The contributions in our paper are as follows:

- To be more comprehensive in our healthcare recommendation system, structural knowledge, textual knowledge, and visual knowledge are involved in the knowledge base.
- The healthcare and medical knowledge graph is leveraged in our system, which can be more precise and accurate.
- A better model can be obtained due to new labelled and processed dataset.
- Deep neural network is utilized in our system to contribute to intelligent various diseases' prediction, diagnosis, and treatment recommendation provided to serve patients and doctors.

The article "Multitask Healthcare Management Recommendation System Leveraging Knowledge Graph" was published in 2021. Journal: J Healthc Eng.

The remainder of this paper is organized as follows: Section 2 introduces the materials and methods which the multimodel healthcare management recommendation system and network architecture and framework contained. In Section 3, the results and discussion are expressed. The paper is concluded in Section 4.

## 2. Materials and Methods

The architecture of our multitask healthcare management recommendation system leveraging the knowledge graph and deep neural network based on 5G network is shown in Figure 1. It can be applied in mobile and terminal device, which is connected to various places, such as hospitals, communities, and homes to integrate users' health information data from multiple channels. The collaborative knowledge graph is input and a multimode knowledge graph entity encoder is utilized in the knowledge graph embedding module. Then the new entity representation is used to learn knowledge graph embedding in order to represent the knowledge inference relationship. In the recommendation module, the embedding was learned by the knowledge graph, also with the collaborative knowledge graph, to enrich the expression of patients and medical items to improve the recommendation effect and the experience. Taking viral pneumonia as an example, when the user passes their data through our system, it will automatically rank the severity of the disease and advise the user on what grade of hospital they should go to and provide other treatment recommendations and so on.

The article "Multitask Healthcare Management Recommendation System Leveraging Knowledge Graph" was published in 2021. Journal: J Healthc Eng.

### 2.1. Multitask Healthcare Management Recommendation System Framework

The framework of our multitask healthcare recommendation is shown in Figure 2, which consists of recommendation task module, feature learning task of the healthcare knowledge graph module, and cross compression unit. In the recommendation part, the feature representation of the user and the item is regarded as input, while the predicted click probability is regarded as output. The features of the user and item are extracted, respectively, by the multilayer perceptron and cross-compression unit and then they are fed into another multilayer perceptron. In the knowledge graph part, the head node of the triple and the relationship representation are considered as input, while the predicted trail node is regarded as output. When a couple of the head and relation is input, the features of the head and relation are also extracted, respectively, by multilayer perceptron and cross-compression unit. Then the representation of predictive tail can be calculated on the basis of the head and the relation; also the similarity between the predicted tail and the actual tail can also be calculated by function *f*. In other words, it is the knowledge graph embedding capability score of the link prediction. However, in practical application, the recommendation task and the feature learning of the knowledge graph are not independent of each other, on account of the overlap between the items in the recommendation system and the entities in the knowledge graph. The cross feature-sharing unit is designed as a connected band between the two tasks, which is the key to connect the recommendation module and the knowledge graph embedding module and can automatically learn the high-level interaction features of recommendation item and knowledge graph entity.

The information can be exchanged in the cross-compression unit in Figure 3. It is seen that the item vector and the entity vector are the two descriptions of the same object actually and the cross-sharing of the information between them allows each to get additional information from each other to make up for the lack of information sparsity. However, it is noted that the cross-compression unit can exist at the lower level of the system. It is known that, along the network, the features can be translated from generic to specific, while the feature transferability is decreased significantly at higher levels with the increased variability in tasks, which can lead to a negative shift in the high-level sharing, especially the heterogeneous task. Besides, in the high layer, the mixed features of item, user, entity, and relation are not suitable for sharing due to none being explicitly related.

The article "Multitask Healthcare Management Recommendation System Leveraging Knowledge Graph" was published in 2021. Journal: J Healthc Eng.

### 2.2. Structural Knowledge

As shown in Figure 4, our healthcare knowledge graph is constructed of various entities and links, which can be considered as a heterogeneous network. Our healthcare knowledge graph model is based on 600 thousand pieces of training data, which has a good performance on department classification, food and drug recommendation, treatment recommendation, and major item examination according to the disease. While this representation method works well for the structured data, it is difficult to process the healthcare knowledge graph. Therefore, the knowledge graph embedding approach is utilized to address the above problem, especially the embedded components, which not only can transform the relationships between entities into a continuous vector space to simply the operation but also can retrain the original structure of the knowledge graph. In our system, the translation distance model is adopted as the knowledge embedding method, in which the distance-based scoring function is utilized and the reasonableness of a fact is measured by the distance between two entities. In general, there are several types of translation distance models including TransE, TransH, TransD, and TransR. It is known that an entity is a complex of properties and different attributes of the entity are focused on by different relationships. In our work, TransD shown in Figure 5, which is the improvement of TransR, is used and it is considered that different entities should be mapped into different semantic spaces. Also, it overcomes the shortcomings of computational complexity and model parameter. Owing to fewer parameters and no matrix vector multiplication in TransD, it can be suitable for our large-scale healthcare knowledge graph.

Two vectors were used to represent each entity and relationship in TransD, and the two mapping matrices are defined as formulas (1) and (2), where the first vector represents the meaning of the entity or relationship and the second vector would be utilized to construct the mapping matrix. It is found that the mapping matrix is defined by entities and relations and *I* represents the identity matrix. In formulas (3) and (4), it is seen that *h*_⊥_ and *t*_⊥_ are projected vectors of entities. The loss function of knowledge representation and training method is shown in formula (6) and the function of *f*_*r*_ is defined in formula (5).

(1) $$\begin{array}{c} M_{rh}=r_{p\;}h_{p}^{T}\;+\;I, \end{array}$$

(2) $$\begin{array}{c} M_{rt}=r_{p\;}t_{p\;}^{T}\;+I, \end{array}$$

(3) $$\begin{array}{c} h_{⊥\;}=\;M_{rh}h, \end{array}$$

(4) $$\begin{array}{c} t_{⊥\;}=\;M_{rt}t, \end{array}$$

(5) $$\begin{array}{c} f_{r\;}\left(h,t\right)\;=\;{\left\|h_{⊥\;}+r\;-t_{⊥\;}\right\|}_{2}^{2}, \end{array}$$

(6) $$\begin{array}{c} L=\underset{\left(h,r,t\right)\in S}{\sum }\underset{\left(h^{\prime },r,t^{\prime }\right)\in S^{\prime }}{\sum }\text{max}\left(0,f_{r}\left(h,t\right)+\gamma -f_{r}\left(h^{\prime },t^{\prime }\right)\right). \end{array}$$

The article "Multitask Healthcare Management Recommendation System Leveraging Knowledge Graph" was published in 2021. Journal: J Healthc Eng.

### 2.3. Textual Knowledge

In our healthcare management system, a large amount of text data on symptoms would be recorded and updated every day. Therefore, the textual knowledge can contribute to the accuracy and efficiency of the analysis of the symptoms and text representation is of great significance, which can convert the symbols of human language into numbers that the machines can compute. In our work, word embedding method of Word2Vec is adopted, which is one of the most commonly used word embedding models and neural network models. Besides, the semantic information of the word can be represented in the form of word vector, and semantically similar words are close together in the space through an embedded space. The word embedding method utilized is shown in Figure 6 and it is similar to the idea of autoencoder. It is constructed based on the training data and then the model learned parameters can be obtained. It is shown that *w*(*t*) is the input word and in the hidden layer it can perform the dot product between matrix and the input vector *w*(*t*) and then the outcome is passed to the output layer. In the output layer, it can calculate the dot product between the output vector of the hidden layer and the weight matrix of the output layer. Then the activation function of softmax is used to calculate the probability that a word appears in the context of *w*(*t*) at a given context location. Finally, Skip-Thought method is utilized as a sentence vector to acquire the textual features representation, which is the encoder-decoder architecture and the GRU model. There are several advantages in Word2Vec and Skip-Thought adopted in our system. Firstly, it can be suitable for any medical and healthcare original text to complete modeling of the relationships between sentences, since it is an unsupervised learning technique. Secondly, it takes less memory which can be applied in mobile terminal device. Finally, it has fewer dimensions in the weight matrix, which leads to fewer computation, which can be fit for healthcare management application.

The probability is shown in formula (7), where *w*(*c*, *j*) represents the predicted *j* word at the *c* context location, *w*(*O*, *c*) represents the actual word that appears at the *c* context position, *w*(*I*) represents the only input word, and *u*(*c*, *j*) represents the *j* value of the *U* vector when a word is predicted at the *c* context position. The loss function is expressed in formula (8), where the probability can be maximized when predicting *w*(*c*, *j*) at the *c* context position.

(7) $$\begin{array}{c} p\left(w_{c,j}=w_{O,c}\;|\;w_{I}\right)=\frac{\text{exp }u_{c,j}}{\sum_{j-1}^{V}\text{exp }u_{j}}, \end{array}$$

(8) $$\begin{array}{c} L=-\text{log }P\left(w_{c,1},w_{c,2},\ldots ,w_{c,C}\;|\;w_{o}\right)=-\sum_{c=1}^{C}u_{c,j^{*}}+\sum_{c=1}^{C}\text{log}\sum_{j=1}^{V}\text{exp}\left(u_{c,j}\right). \end{array}$$

The article "Multitask Healthcare Management Recommendation System Leveraging Knowledge Graph" was published in 2021. Journal: J Healthc Eng.

### 2.4. Visual Knowledge

It is demonstrated that visual knowledge also plays an important role in our healthcare management recommendation system; and there are many diseases that need medical images to perform further diagnosis, for example, lung disease, liver disease, and femoral head disease. In our healthcare management system, a large number of medical images also would be uploaded and updated. In order to obtain the semantic information and the embedded representation of the image, the backbone network ResNet would be adopted in our system. The structure of the residual learning block is shown in Figure 7. It is obvious that ResNet is a residual network which can be stacked to form a deep network, which contains a natural identity mapping that can solve the problem of network degradation to some extent. What is more, the mapping with residuals is more sensitive to changes in output. Also, in forward propagation, the input signal can propagate directly from any low level to the high level and error signals can be propagated directly to the lower level without any intermediate weight matrix transformation. Therefore, to some degree, the problem of gradient dispersion can be alleviated, which allows information to propagate back and forth more smoothly in residual connection. The residual unit is expressed in formula (9), where *x*_*l*_ and *x*_*l*+1_ represent the input and the output of the residual unit of *l*, respectively. In addition, *F* is the residual function, which represents the learned residual and *h* (*x*_l_) represents the identity mapping. In formula (10), *f* is the ReLU activation function. The learning feature from shallow layer *l* to deep layer *L* is expressed in formula (11). The gradient of the reversed process can be obtained by the chain rule in formula (12), where 1 shows that the short-cut mechanism can propagate the gradient without loss and in the other item the residual gradient passes through a layer with weights.


(9) $$\begin{array}{c} y_{l}\;=\;h\left(x_{l}\right)\;+F\left(x_{l},\;W_{l}\right), \end{array}$$

(10) $$\begin{array}{c} x_{l+1}\;=\;f\left(y_{l}\right), \end{array}$$

(11) $$\begin{array}{c} x_{L}\;=\;x_{l}\sum_{i=1}^{L-1}F\left(x_{i},W_{I}\right), \end{array}$$

(12) $$\begin{array}{c} \frac{\partial \text{loss}}{\partial x_{L}}=\frac{\partial \text{loss}}{\partial x_{l}}\cdot \frac{\partial \text{loss}}{\partial x_{L}}=\frac{\partial \text{loss}}{\partial x_{L}}\cdot \left(1+\;\frac{\partial }{\partial x_{L}}\sum_{i=1}^{L-1}F\left(x_{i},W_{i}\right)\right). \end{array}$$

The architecture of the backbone network ResNet is shown in Figure 8, in which each residual block can constitute a residual network and convolution layer, Batchnorm, ReLU, Maxpool, Convblock, IDblock, and so on involved to acquire the medical images representation. The ID block (Identity block) is shown in Figure 9 and the convolutional block is shown in Figure 10.

The article "Multitask Healthcare Management Recommendation System Leveraging Knowledge Graph" was published in 2021. Journal: J Healthc Eng.

### 2.5. Healthcare Management Knowledge Graph Encoder

Our multitask healthcare knowledge graph encoder is shown in Figure 11. The healthcare structural knowledge was embedded by translation distance model TransD, the healthcare textual knowledge was embedded by word embedding method Word2Vec and a sentence vector Skip-Thought method to acquire the textual features representation, and the visual knowledge was embedded by ResNet backbone network to obtain the semantic information and the embedded representation of the image. They were regarded as tail to be input, and then they passed through the dense layer to make the features extracted above nonlinearly changed to acquire the correlation between these features and then mapped to the output space to obtain the dense vector.

The loss function of our healthcare management system is shown in formula (13), where the first term is the cross-entropy loss of the recommendation module and *u* and *v* are the the users and items collections which have been traversed. What is more, the second term is the loss of knowledge graph embedding module, the aim of which is to increase the score of the correct triple and reduce the score of the error triples. In addition, the third item is regular item to prevent overfitting, where *λ*_1_ and *λ*_2_ are the equilibrium constants.

(13) $$\begin{array}{c} L=L_{\text{RS}}+L_{\text{KG}}+L_{\text{REG}}\\ =\underset{u\in U,v\in V}{\sum }ℐ\left({\hat{y}}_{uv},y_{uv}\right)-\lambda_{1}\left(\underset{\left(h,r,t\right)\in G}{\sum }\text{score}\left(h,r,t\right)-\underset{\left(h^{\prime },r,t^{\prime }\notin G\right)}{\sum }\text{score}\left(h^{\prime },r,t^{\prime }\right)+\lambda_{2}{\left\|W\right\|}_{2}^{2}\right.. \end{array}$$

The article "Multitask Healthcare Management Recommendation System Leveraging Knowledge Graph" was published in 2021. Journal: J Healthc Eng.

## 3. Results and Discussion

Table 1 shows the recall (state of the art) in different models for our dataset. It is obvious that our multitask healthcare management recommendation system has better performance compared to other common recommendation systems. What is more, compared with base models, our system still performs better than text-based and image-based models in Table 2. The bar chart is shown in Figures 12 and 13. It is seen that our multitask healthcare management recommendation system is encouraging, which is more convenient to serve the patients and doctors to perform disease prediction and provide treatment recommendation. In addition, it can free up and alleviate medical resources to make it balanced in medical field. However, there exist some limitations in this system to recommend the most suitable doctor corresponding to the disease due to lack of the doctors data, which needs to be solved in the future.

## 4. Conclusions

In conclusion, it is shown that our multitask healthcare management recommendation system is intelligent and promising, which can free up and alleviate the medical resources to be more convenient and efficient. In addition, it has advantages compared to other common methods in propagating and generalizing the data to obtain the high-value and useful information for the patients and the doctors. However, due to lack of the doctors data, our system is not able to recommend the appropriate doctor corresponding to the disease. Besides, there are still some limitations in comprehensive professional guidance in our recommendation system. In the future, abundant doctors data should be added and processed, accompanied by more professional guidance to support out healthcare management recommendation system to make it more comprehensive.

## Figures and Tables

**Figure 1:** The architecture of our multitask healthcare management intelligent recommendation system.

**Figure 2:** The framework of multitask healthcare management recommendation system.

**Figure 3:** The cross-compression unit.

**Figure 4:** Healthcare knowledge graph.

**Figure 5:** The illustration of TransD.

**Figure 6:** The architecture of Skip-Gram.

**Figure 7:** The structure of residual learning block.

**Figure 8:** The architecture of ResNet.

**Figure 9:** The architecture of ID block.

**Figure 10:** The architecture of convolutional block.

**Figure 11:** Multitask healthcare knowledge graph encoder.

**Figure 12:** The comparison of recall in different models for our dataset.

**Figure 13:** The comparison of recall in our models and base models for our dataset.

**Table 1:** The comparison of recall (state of the art) in different models for our dataset.

Model	Recall
NFM	0.2595
CKE	0.2719
RippleNet	0.2791
MKR	0.2812
NGCF	0.2819
KGAT	0.2827
MMGCN	0.2979
Ours	0.3126

The article "Multitask Healthcare Management Recommendation System Leveraging Knowledge Graph" was published in 2021. Journal: J Healthc Eng.

**Table 2:** The comparison of recall (state of the art) in our models and base models for our dataset.

Model	Recall
Base	0.0712
Base + image	0.0755
Base + text	0.0729
Ours	0.0771

## Data Availability

The data used are available and can be accessed to perform multitask healthcare management recommendation system based on knowledge graph. Part of the data are available from the corresponding author upon request (liuwanheng301@163.com).
